# Quantifying the Elasticity Properties of the Median Nerve during the Upper Limb Neurodynamic Test 1

**DOI:** 10.1155/2022/3300835

**Published:** 2022-03-20

**Authors:** Ming Lin, Yaodong Chen, Weixin Deng, Hongying Liang, Suiqing Yu, Zhijie Zhang, Chunlong Liu

**Affiliations:** ^1^Clinical Medical College of Acupuncture, Moxibustion and Rehabilitation, Guangzhou University of Chinese Medicine, Guangzhou, China; ^2^Guangzhou University of Chinese Medicine, Guangzhou, China; ^3^Luoyang Orthopedic Hospital of Henan Province, Luoyang, China

## Abstract

**Background:**

The upper limb neurodynamic test 1 (ULNT1) consists of a series of movements that are thought to detect an increase in neuromechanical sensitivity. In vivo, no trail was made to quantify the association between the nerve elasticity and different limb postures during ULNT1.

**Objectives:**

(1) To investigate the relationship between nerve elasticity and limb postures during ULNT1 and (2) to investigate the intra- and interoperator reliabilities of shear wave elastography (SWE) in quantifying the elasticity of median nerve.

**Methods:**

Twenty healthy subjects (mean age: 19.9 ± 1.4 years old) participated in this study. The median nerve was imaged during elbow extension in the following postures: (1) with neutral posture, (2) with wrist extension (WE), (3) with contralateral cervical flexion (CCF), and (4) with both WE and CCF. The intra- and interoperator reliabilities measured by two operators at NP and CCF+WE and intraclass correlation coefficients (ICCs) were calculated.

**Results:**

The intraoperator (ICC = 0.72–0.75) and interoperator (ICC = 0.89–0.94) reliabilities for measuring the elasticity of the median nerve ranged from good to excellent. The mean shear modulus of the median nerve increased by 53.68% from NP to WE+CCF.

**Conclusion:**

SWE is a reliable tool to quantify the elasticity of the median nerve. There was acute modulation in the elasticity of the median nerve during the ULNT1 when healthy participants reported substantial discomfort. Further studies need to focus on the elasticity properties of the median nerve in patients with peripheral neuropathic pain.

## 1. Introduction

The upper limb neurodynamic test 1 (ULNT1) consists of a series of movements constructed to stress various parts of the nervous system and is regarded to be capable of detecting increased nerve mechanosensitivity [1, 2]. Clinicians use range of motion (ROM) and sensory responses to evaluate neurodynamic tests and compare sides and/or relate results to normal values in order to diagnose upper extremity peripheral neuropathic pain [3, 4]. Furthermore, musculoskeletal physiotherapists evaluate ULNT1 (median nerve) to discover changes in mechanosensitivity in the neural system, hence measuring function gain for patients [5]. The ULNT1 is very widely used in clinical settings.

Previous research has combined ULNT1 with psychological questionnaires such as the visual analogue scale (VAS) to assess prognosis and treatment response [6, 7]. However, these psychological surveys are unable to rule out the effects of placebos, cognitive, and other psychophysiological alterations. Researchers were expected to establish a more objective reference standard for peripheral neuropathic pain in order to validate the efficacy of ULNT1 [8]. The biomechanics of neurodynamic studies in vitro may be characterized by a combination of stress, strain, and movement [9]. According to a systematic review of research [10], frame-by-frame cross-correlation software was utilized to detect nerve motion in all trials. Limb movement induces complex biomechanical effects such as nerve elongation, nerve longitudinal and transverse excursion, and changes in diameter [9, 10]. These trials are performed using ultrasound techniques to detect nerve displacement while changing joint posture and lack the detection of nerve stress (tension) in vivo. In addition, the ultrasonographer measured the displacement and cross-sectional area of nerve movements by hand, and the measurement's reliability (ICC = 0.542) was determined by the ultrasonographer's own experience [11]. The displacement is insensitive to the nerve's tissue stress. A suitable instrument with adequate properties was not available. Therefore, it is necessary to seek a device that can detect stress to standardize the neurophysiological stress range in vivo.

In recent years, shear wave elastography (SWE) technology has produced a measurable depiction of “elasticity” in tissues [12–14]. Hooke's law, which establishes the relationship between strain, stress, and elasticity only in isotropic and purely elastic media, is the foundation of SWE: *s* = *E* · *d* (*E*: elasticity; *s*: stress; and *d*: strain) [15]. Elasticity is defined as the ratio of stress to strain, which reflects the structural stress of tissue indirectly [16]. The biomechanical parameter used to characterize elasticity is the shear modulus. However, there are few trials using SWE devices to assess the elastic properties of the nerves. There is no consensus on the physiological parameters of neuroelasticity. To the authors' knowledge, SWE has not been used to observe the modulation of elasticity in the median nerve during ULNT1. It is necessary to validate the repeatability of the SWE technique applied to nerve elasticity detection in ULNT1.

Therefore, the goals of this study were to (1) assess the reliability of SWE in quantifying the elasticity of the median nerve and (2) analyze the elasticity modifications of the median nerve among four variations of ULNT1.

## 2. Materials and Methods

### 2.1. Ethics Statement

The Ethics Committee of Guangdong Provincial Hospital of Traditional Chinese Medicine (YE2020-329-01) authorized all procedures for this study, which was conducted out in accordance with the Helsinki Declaration. The goal of the study was clearly disclosed to all subjects. The experimental protocols and the safety of SWE were explained in detail in the experimental statement, and each participant completed an informed permission form.

### 2.2. Subjects

Twenty healthy college students (7 males and 13 females; age: 19.9 ± 1.4 years) were recruited in this study: height: 165.00 ± 6.75 cm and weight: 54.07 ± 6.85 kg. Healthy subjects did not have any indication of nerve involvement and were excluded if they presented a history of systemic neurological disorders, posttraumatic changes to the nerve, nerve tumors, nerve entrapment syndromes, musculoskeletal disorders, or other systemic metabolic diseases.

### 2.3. Equipment

All elastography examinations were performed by the ultrasound SWE system (Aixplorer Supersonic Imagine, France) with a 4–15 MHz and 40 mm linear transducer. Other settings of the SWE systems were as follows for best image quality: The opacity was 85% in the musculoskeletal mode, and the depth of the B-scan ultrasound was 2.5 cm. The diameter of the regions of interest (ROIs) was adjusted to 2 mm. The color scale ranged from 0 to 600 kPa. The change is from blue (soft) to red (hard) based on the shear modulus.

### 2.4. Procedure

The subjects sit upright on a chair with their upper arms positioned horizontally, with the shoulder abducted 90 degrees and 90 degrees externally rotated. There are no relevant studies to prove that lower extremity joint movements affect the elasticity of the upper extremity nerves. Their arms were supported by the table, relaxed, and extended toward the experimenter. Keep the fingers still to avoid nerve displacement caused by other joint movements [17]. An adjustable aluminum head restraint was positioned against the side of the head in the temporal region to adjust the contralateral cervical flexion angle. An adjustable wrist hand splint was designed to maintain the hand and wrist passively in the chosen position. When the participant reported substantial discomfort, the maximum angle of the extended wrist in the cervical neutral position and the maximum angle of contralateral cervical flexion in the wrist neutral position were recorded, respectively, with 5 min of rest between the different variants (see Figure 1).

Elasticity measurement was performed 30 minutes after the angle measurement. The elasticity measurement was positioned at the midpoint of the forearm (from transverse wrist to transverse elbow). Light pressure was defined as placing the transducer lightly on top of a generous amount of coupling agents on the skin [18]. Nerves were verified in the transverse plane by the honeycomblike structure. The transverse imaging plane of the nerve was identified by B-mode. Then, the transducer was rotated 90° to obtain the longitudinal imaging plane, which was a parallel orientation to the nerve. The transducer remained stationary for more than 5 seconds until the color in the ROI was uniform. The image was frozen and placed in the Q-box to obtain the shear modulus. The shear modulus of the median nerve was measured in 4 variants of the upper limb neurodynamic test 1, which included the following positions: (1) neutral posture (NP), (2) wrist extension (WE), (3) contralateral cervical flexion (CCF), and (4) both wrist extension and contralateral cervical flexion (WE+CCF), with a 3-minute rest between each measurement. The mean of three values in each measurement was used for further analysis.

Repeatability was assessed by measuring SWE of the median at the NP and WE+CCF. Operator A and operator B participated in the interoperability survey. Two operators (A and B), both trained in SWE, conducted the full examinations, respectively. The operators took turns examining each subject's median nerve over a 1-hour period and by operator B with a 2-hour interval (test 1st). Five days after the first measurement, the same subject was rechecked by operator A (test 2nd), and the shear modulus was used to calculate the intraoperator repeatability. Twenty healthy people were chosen at random to be tested for inter- and intraoperator reliability. The two operators were blinded to the results.

### 2.5. Statistical Analysis

Statistical analysis was performed using SPSS 18.0 software (SPSS Inc., Chicago, IL, USA). The Shapiro-Wilk test was used to check the normal distribution of all stiffness data. The mean ± standard deviation was used to express all stiffness data. A one-way repeated measures analysis of variance (ANOVA) was used to compare the variability of the shear modulus of the four variants of the ULNT1. Multiple comparisons were accounted for by using Bonferroni corrections. The intra- and interoperator reliabilities were calculated using the intraclass correlation coefficient (ICC) and a 95% confidence interval. The ICC (3,1) (two-way mixed-effect model, consistency) was obtained to evaluate the agreement between the two tests for operator A. The ICC (2,2) (two-way random effects model, absolute agreement) was obtained to evaluate the agreement between operator A and operator B. The standard error measurement (SEM) was calculated based on the following formula: SEM = standard deviation × √1 − ICC. The minimal detectable change (MDC) was computed using the following formula: MDC = 1.96 × SEM × √2. The Bland-Altman plots further intuitively indicated the degree of consistency in assessing intra- and interoperator reliabilities, in which the *x*-axis represented the average [(K1 + K2)/2] and the *y*-axis represented the difference (K1–K2) of the two measurements. The ICC was classified as poor (0.00–0.20), fair (0.21–0.40), good (0.41–0.75), or excellent (>0.75) [19]. The statistical significance level was set an alpha level of *p* < 0.05 (*α* = 0.05).

## 3. Results

### 3.1. Intra- and Interoperator Reliabilities

The intra- and interoperator reliabilities of shear modulus of the median nerve is presented in Table 1. The ICC values reveal good intraoperator reliabilities at NP (ICC = 0.75; 95% CI = 0.58–0.86; SEM = 10.54 kPa; and MDC = 29.21 kPa) and CCF+WE (ICC = 0.72; 95% CI = 0.53–0.84; SEM = 33.19 kPa; and MDC = 91.99 kPa). The ICC values reveal excellent interoperator reliabilities at NP (ICC = 0.94; 95% CI = 0.90–0.97; SEM = 5.44 kPa; and MDC = 15.07 kPa) and CCF+WE (ICC = 0.89; 95% CI = 0.79–0.94; SEM = 20.64 kPa; and MDC = 57.21 kPa). The Bland-Altman plot for reliability of SWE measurement between 5 days at NP and CCF+WE is presented in Figures 2(a) and 3(a). The Bland-Altman plot for reliability of SWE measurement between two operators at NP and CCF+WE is shown in Figures 2(b) and 3(b).

### 3.2. Changes in Median Nerve during ULNT1

The mean shear modulus of the median nerve in the middle forearm was 137.71 ± 22.72 kPa at the neutral posture, only contralateral cervical flexion was 211.00 ± 30.49 kPa, and only wrist extension was 252.34 ± 40.30 kPa and 297.35 ± 64.60 kPa at contralateral cervical flexion+wrist extension (see Figure 4). The mean shear modulus of the median nerve increased by 53.68% from neutral position to contralateral cervical flexion+wrist extension.

## 4. Discussion

This study was to investigate the modulation of the shear modulus of the median nerve at the midpoint of the forearm during ULNT1. The main findings of this study were that SWE has good to excellent intra- and interoperator reliabilities in quantifying the shear modulus of the median nerve. When the participant reports substantial discomfort, there were differences in the shear modulus of the median nerve in different joint variations.

### 4.1. Intra- and Interoperator Reliabilities

The intraoperator reliabilities (ICC = 0.72 − 0.75) in quantifying the median nerve elasticity by SWE at NP and CCF+WE were good. The interoperator reliabilities (ICC = 0.89 − 0.94) in quantifying the median nerve elasticity by SWE at NP and CCF+WE were excellent. SWE is a reliable and reproducible noninvasive method for the assessment of tissue elasticity [20, 21]. According to one research, the ICC of interobserver measures of liver elasticity on several dates was 0.84 [20]. The interoperator and intraoperator reliabilities for measuring median nerve elasticity by SWE were excellent (ICC: 0.852-0.930), according to Zhu et al. [21]. However, operators must be well trained; the ICC of unskilled testers was just 0.65 [22]. In conclusion, SWE is a noninvasive and acceptable tool for quantifying the elasticity of the median nerve during ULNT1.

In the current study, the ICC values for interoperator reliabilities in NP (ICC = 0.94) and CCF+WE (ICC = 0.89) were relatively high compared to the ICC values for intraoperator reliabilities in NP (ICC = 0.75) and CCF+WE (ICC = 0.72). We considered that the operator measured elastography at an interval of 5 days. The subjects are unavoidably engaged in a variety of activities that strained the nerve tissue. It might have an effect on the nerve's biomechanical structure. The ICC values for neutral posture might have been higher than those for contralateral cervical flexion+wrist extension. Nerve tissue, like other soft tissues, has complicated viscoelastic and creeping properties. Neck flexion and wrist extension were done at the same time. Because the nerve tissue had been stretched, severe mechanical stresses were more likely to cause creeping behavior. The Bland-Altman plot provides visual evaluation for limits of agreement. Almost all the points that were included in the 95% confidence interval were shown in Figures 2 and 3, which indicates that the intra- and interoperator reliabilities have high consistency at NP. Besides, an ideal agreement is zero difference between two measurements [23]. The Bland-Altman plots of interoperator (Mean = 2.0) has smaller mean difference than the intraoperators' (Mean = 4.5) in NP. The Bland-Altman plots of interoperator (Mean = 5.2) has smaller mean difference than the intraoperators' (Mean = 6.8) in CCF+WE. In the present study, two operators underwent training prior to the experiment, which included the anatomy of the tissue investigated, basic biomechanical concepts of the tissue, and the limitations of the SWE tool. So two operators were measuring in a way that met the SWE guideline. SWE uses an acoustic radiation force impulse, which does not require specific experience of the examiner and contributes to the consistent reliability [15]. As a result, the Bland-Altman plots further verified the reliability of our study data.

In this study, we also calculated the MDC of neutral posture; the MDC provides an objective threshold that can be used to determine whether values obtained are beyond measurement variability. Our study results showed that the MDC of the median nerve was 29.21 kPa (the same operator) and 15.07 kPa (different operator). Therefore, the shear modulus of the median nerve should be larger than 15.07 kPa to reflect changes with retested tests.

### 4.2. Immediate Alterations of Median Nerve of Joint Rotation

According to the findings of the current investigation, the shear modulus of the median nerve at neutral posture was 137.71 kPa. At the CCF, this value climbed to 211.00 kPa. The median nerve's shear modulus rose by 34.73%. The structure of peripheral nerves offers significant adaptability for joint mobility due to the continuity of the complete body's neural system [24]. The current study found that the elasticity of the median nerve at the forearm's midpoint may be modulated in vivo during cervical lateral flexion. The length of the nerve bed varies in response to joint movement [25, 26]. The longitudinal displacement of the median nerve in the forearm was 2.3 mm when cervical lateral flexion was applied [27]. Movement of the joint can modify the elasticity property of the median nerve when enough mechanical stress is applied to it [28, 29].

The results have shown that the shear modulus of the median nerve was 252.34 ± 40.30 kPa at only wrist extension. From NP to WE, the shear modulus of the median nerve increased by 46.21%. When subjects reported substantial discomfort, the shear modulus of the median nerve was higher in WE than in CCF. One explanation was the anatomical location of the median nerve. The median nerve was squeezed by the wrist flexors during wrist extension [30]. The superimposed action of squeezing increased the nerve's shear modulus. No changes in strain or excursion of the flexor digitorum superficialis are caused by neck movement [31]. Another argument was that the subject's discomfort was not caused by the nerves being stretched. The pain might be coming from the muscles or the skin being stretched.

Furthermore, the total of WE and CCF was greater than the shear modulus of WE+CCF. Complex viscoelastic behavior is observed in nerve tissues. During movement, peripheral nerves are put under mechanical stress of skeletal muscle. First, the consistent tissue structure of the median nerve might justify this variance [32, 33], which has greater folded torsion at the joint. Second, consider the possibility of a cause in the soft tissue relaxation stress curve. There is a crucial strain associated with each fiber tissue (corresponding to its length). The nerve fibers change their elasticity only when they are taut [34]. No more elastic strain occurred when the extension reached a yield point. As a result, even within the physiological range of joint motion, simultaneous movement of the extremities should not be too rapid.

SWE can be used to investigate the elasticity property of the median nerve. In addition, neural mobilization was based on the anatomical structure, physiological functions, and neurodynamics of the peripheral nervous system [35, 36]. Neurodynamic assessments developed into nerve mobilization for therapeutic rehabilitation applications. Neto et al. [37] observed that following nerve mobilization, the shear modulus of the sciatic nerve was lowered by 16.1% in individuals with sciatica. Driscoll et al. [38] showed that applying suitable mechanical stress might increase the blood circulation of ascending and descending branches of nutrition arteries on the neuron connective tissue membrane, hence improving nerve function and promoting rehabilitation.

## 5. Limitations

This study does have some limitations. First, in a healthy young person, the shear modulus of the median nerve was not fully constant. Other factors' influence on neural characteristics were not investigated. Second, this study only looked at the elasticity of the median nerve in healthy individuals. It was hard to foresee whether the surgery would worsen the clinical symptoms of peripheral nerve disease patients. Further study will be done on the repeatability of individuals with peripheral nerve disease. Finally, the sample size of subjects in this study was relatively small. The next study will collect a large sample to determine the elasticity range of the median nerve, which would help to identify the pathological elasticity of the nerve in a clinical setting.

## 6. Conclusion

SWE has the potential to be a viable instrument for measuring the elastic properties of the median nerve during ULNT1. The elasticity of the median nerve in the forearm changed during ULNT1 when healthy volunteers felt substantial discomfort. Shear modulus can provide a quantitative indicator of the physiological structure of nerve. It also can be a straightforward and easy therapy for primary care patients.

## Figures and Tables

**Figure 1:** Schematic diagram of upper limb neurodynamic testing. Images of the median nerve between the superficial flexor and the deep flexor at the midpoint of the forearm which is sampled and measured; the color area of the image is the elastic image area of shear wave and the measured area neutral posture (a); contralateral cervical flexion (b); wrist extension (c); and contralateral cervical flexion+wrist extension (d).

**Figure 2:** Bland-Altman plots of intra- and interoperator reliabilities for the shear modulus of the median nerve in the neutral posture (NP). Intraoperator reliability (a): the difference in median nerve stiffness between day 1 and day 5 is plotted against mean median nerve stiffness (average of the 2 days for operator A) for each subject. Interoperator reliability (b): the difference in median nerve stiffness between operator A and operator B is plotted against mean median nerve stiffness (average of the 2 operators) for each subject. The continuous lines represent the mean difference, while the dotted lines show the 95% upper and lower limits of agreement.

**Figure 3:** Bland-Altman plots of intra- and interoperator reliabilities for the shear modulus of the median nerve in the contralateral cervical flexion+wrist extension (CCF+WE). Intraoperator reliability (a): the difference in median nerve stiffness between day 1 and day 5 is plotted against mean median nerve stiffness (average of the 2 days for operator A) for each subject. Interoperator reliability (b): the difference in median nerve stiffness between operator A and operator B is plotted against mean median nerve stiffness (average of the 2 operators) for each subject. The continuous lines represent the mean difference, while the dotted lines show the 95% upper and lower limits of agreement.

**Figure 4:** Box plot of the shear modulus of the median nerve at the midpoint of the forearm for 4 variants of the upper limb neurodynamic test (black: neutral posture (NP); dark gray: contralateral cervical flexion (CCF); light gray: wrist extension (WE); white: contralateral cervical flexion+wrist extension (CCF+WE)). ∗∗ indicates *p* < 0.001.

**Table 1:** Intra- and interoperator reliabilities of SWE for assessing the shear modulus of the median nerve.

	Variant	Test 1st (kPa)	Test 2nd (kPa)	95% CI	SEM (kPa)	MDC (kPa)	ICC
Intraoperator reliability	NP	137.71 ± 22.72	142.23 ± 21.08	0.58–0.86	10.54	29.21	0.75
	CCF+WE	297.35 ± 64.60	290.58 ± 62.73	0.53–0.84	33.19	91.99	0.72

		Operator A	Operator B	95% CI	SEM	MDC	ICC
Interoperator reliability	NP	137.71 ± 22.72	135.70 ± 22.21	0.90–0.97	5.44	15.07	0.94
	CCF+WE	297.35 ± 64.60	292.11 ± 62.25	0.79–0.94	20.64	57.21	0.89

ICC: intraclass correlation coefficient; CI: confidence interval; SEM (kPa): standard error of measurement of kPa; MDC (kPa): minimal detectable change; SD (kPa): standard deviation of kPa; kPa: kilo Pascal; NP: neutral posture; CCF+WE: contralateral cervical flexion+wrist extension.

## Data Availability

All data included in this study are available upon request by contact with the corresponding author.

## References

[1] Koulidis K., Veremis Y., Anderson C., Heneghan N. R. (2019). Diagnostic accuracy of upper limb neurodynamic tests for the assessment of peripheral neuropathic pain: a systematic review. *Musculoskeletal Science & Practice*.

[2] Riley S. P., Grimes J. K., Calandra K., Foster K., Peet M., Walsh M. T. (2020). Agreement and reliability of median neurodynamic test 1 and resting scapular position. *Journal of Chiropractic Medicine*.

[3] Grondin F., Cook C., Hall T., Maillard O., Perdrix Y., Freppel S. (2021). Diagnostic accuracy of upper limb neurodynamic tests in the diagnosis of cervical radiculopathy. *Musculoskeletal Science & Practice*.

[4] Trillos M. C., Soto F., Briceno-Ayala L. (2018). Upper limb neurodynamic test 1 in patients with clinical diagnosis of carpal tunnel syndrome: a diagnostic accuracy study. *Journal of Hand Therapy*.

[5] Baselgia L. T., Bennett D. L., Silbiger R. M., Schmid A. B. (2017). Negative neurodynamic tests do not exclude neural dysfunction in patients with entrapment neuropathies. *Archives of Physical Medicine and Rehabilitation*.

[6] Whelan G., Johnston R., Millward C., Edwards D. J. (2018). The immediate effect of osteopathic cervical spine mobilization on median nerve mechanosensitivity: a triple-blind, randomized, placebo-controlled trial. *Journal of Bodywork and Movement Therapies*.

[7] Calvo-Lobo C., Unda-Solano F., López-López D. (2018). Is pharmacologic treatment better than neural mobilization for cervicobrachial pain? A randomized clinical trial. *International Journal of Medical Sciences*.

[8] Nee J., Jull G. A., Vicenzino B., Coppieters M. W. (2012). The validity of upper-limb neurodynamic tests for detecting peripheral neuropathic pain. *The Journal of Orthopaedic and Sports Physical Therapy*.

[9] Topp K. S., Benjamin S. B. (2006). Structure and biomechanics of peripheral nerves: nerve responses to physical stresses and implications for physical therapist practice. *Physical Therapy*.

[10] Szikszay T. H., von Piekartz H. (2017). In vivo effects of limb movement on nerve stretch, strain, and tension: a systematic review. *Journal of Back and Musculoskeletal Rehabilitation*.

[11] Cornelson M., Sclocco R., Kettner N. W. (2019). Ulnar nerve instability in the cubital tunnel of asymptomatic volunteers. *Journal of Ultrasound*.

[12] Park E. J., Hahn S., Yi J., Shin K. J., Lee Y., Lee H. J. (2021). Comparison of the diagnostic performance of strain elastography and shear wave elastography for the diagnosis of carpal tunnel syndrome. *Journal of Ultrasound in Medicine*.

[13] He Y., Xiang X., Zhu B. H., Qiu L. (2019). Shear wave elastography evaluation of the median and tibial nerve in diabetic peripheral neuropathy. *Quantitative Imaging in Medicine and Surgery*.

[14] Paluch Ł., Noszczyk B., Nitek Ż., Walecki J., Osiak K., Pietruski P. (2018). Shear-wave elastography: a new potential method to diagnose ulnar neuropathy at the elbow. *European Radiology*.

[15] Creze M., Nordez A., Soubeyrand M., Rocher L., Maître X., Bellin M. F. (2018). Shear wave sonoelastography of skeletal muscle: basic principles, biomechanical concepts, clinical applications, and future perspectives. *Skeletal Radiology*.

[16] Hall J. (2003). AAPM/RSNA physics tutorial for residents: topics in US: beyond the basics: elasticity imaging with US. *Radiographics*.

[17] Woo H. C., White P., Ng H. K., Lai C. W. (2016). Development of kinematic graphs of median nerve during active finger motion: implications of smartphone use. *PloS one*.

[18] Strakowski J. A. (2016). Ultrasound-guided peripheral nerve procedures. *Physical Medicine and Rehabilitation Clinics of North America*.

[19] Miyamoto H., Halpern E. J., Kastlunger M. (2014). Carpal tunnel syndrome: diagnosis by means of median nerve elasticity--improved diagnostic accuracy of US with sonoelastography. *Radiology*.

[20] Ferraioli G., Tinelli C., Zicchetti M. (2012). Reproducibility of real-time shear wave elastography in the evaluation of liver elasticity. *European Journal of Radiology*.

[21] Zhu B., Yan F., He Y. (2018). Evaluation of the healthy median nerve elasticity: feasibility and reliability of shear wave elastography. *Medicine*.

[22] Ferraioli G., Tinelli C., Lissandrin R. (2014). Ultrasound point shear wave elastography assessment of liver and spleen stiffness: effect of training on repeatability of measurements. *European Radiology*.

[23] Doğan N. Ö. (2018). Bland-Altman analysis: a paradigm to understand correlation and agreement. *Turkish journal of emergency medicine*.

[24] Brown J. M., Yablon C. M., Morag Y., Brandon C. J., Jacobson J. A. (2016). US of the peripheral nerves of the upper extremity: a landmark approach. *Radiographics*.

[25] Coppieters M. W., Alshami A. M. (2007). Longitudinal excursion and strain in the median nerve during novel nerve gliding exercises for carpal tunnel syndrome. *Journal of Orthopaedic Research*.

[26] Silva A., Manso A., Andrade R., Domingues V., Brandão M. P., Silva A. G. (2014). Quantitative in vivo longitudinal nerve excursion and strain in response to joint movement: a systematic literature review. *Clinical Biomechanics (Bristol, Avon)*.

[27] Brochwicz P., von Piekartz H., Zalpour C. (2013). Sonography assessment of the median nerve during cervical lateral glide and lateral flexion. Is there a difference in neurodynamics of asymptomatic people?. *Manual Therapy*.

[28] Kerns J., Piponov H., Helder C., Amirouche F., Solitro G., Gonzalez M. (2019). Mechanical properties of the human tibial and peroneal nerves following stretch with histological correlations. *Anatomical Record*.

[29] Mahan M. A., Yeoh S., Monson K., Light A. (2019). Rapid stretch injury to peripheral nerves: biomechanical results. *Neurosurgery*.

[30] Behrens M., Husmann F., Mau-Moeller A., Schlegel J., Reuter E. M., Zschorlich V. R. (2019). Neuromuscular properties of the human wrist flexors as a function of the wrist joint angle. *Frontiers in bioengineering and biotechnology*.

[31] Bueno-Gracia E., Pérez-Bellmunt A., Estébanez-de-Miguel E. (2020). Effect of cervical contralateral lateral flexion on displacement and strain in the median nerve and flexor digitorum superficialis at the wrist during the ULNT1 - Cadaveric study. *Musculoskeletal science & practice*.

[32] Jenny C., Lütschg J., Broser P. J. (2020). Change in cross-sectional area of the median nerve with age in neonates, infants and children analyzed by high-resolution ultrasound imaging. *European Journal of Paediatric Neurology*.

[33] Billakota D. S., Ruch D. S., Hobson-Webb L. D. (2018). Ultrasound imaging of median nerve conduit in a patient with persistent median nerve symptoms. *Journal of Clinical Neurophysiology*.

[34] Shearer W., Parnell J., Lynch B., Screen H. R. C., David Abrahams I. (2020). A recruitment model of tendon viscoelasticity that incorporates fibril creep and explains strain-dependent relaxation. *Journal of biomechanical engineering*.

[35] Basson A., Olivier B., Ellis R., Coppieters M., Stewart A., Mudzi W. (2017). The effectiveness of neural mobilization for neuromusculoskeletal conditions: a systematic review and meta-analysis. *The Journal of Orthopaedic and Sports Physical Therapy*.

[36] Basson A., Olivier B., Ellis R., Coppieters M., Stewart A., Mudzi W. (2015). The effectiveness of neural mobilizations in the treatment of musculoskeletal conditions: a systematic review protocol. *JBI Database of Systematic Reviews and Implementation Reports*.

[37] Neto T., Freitas S. R., Andrade R. J. (2020). Shear wave elastographic investigation of the immediate effects of slump neurodynamics in people with sciatica. *Journal of Ultrasound in Medicine*.

[38] Driscoll P. J., Glasby M. A., Lawson G. M. (2002). An in vivo study of peripheral nerves in continuity: biomechanical and physiological responses to elongation. *Journal of Orthopaedic Research*.

